# Stent Applications for Palliative Treatment in Advanced Stage Esophageal Cancers

**DOI:** 10.1155/2021/8034948

**Published:** 2021-10-18

**Authors:** Mustafa Şentürk, Murat Çakır, Mehmet Aykut Yıldırım, Ömer Kişi

**Affiliations:** Department of General Surgery, Necmettin Erbakan University Meram Medicine Faculty, Turkey

## Abstract

**Methods:**

We examined cases of endoscopic stenting for palliative treatment of advanced stage esophageal cancers between January 2014 and July 2019. Age, gender, location of mass, adverse events, survival time, and stent type were evaluated. Outcomes of fully covered and uncovered self-expanding stents were compared with regard to adverse events, including stent migration and occlusion.

**Results:**

The mean age of the patients was 66.4 ± 1, 52 were male, and 8 were female. Patients were followed up for a mean of 133 days. The most common complication due to stenting was migration. 13 patients developed adverse events. Migration was the most common adverse event, occurring in 8 (13%) patients. Although the migration rate of fully covered stents was higher than uncovered stents, there was no statistically significant difference (*p* = 0.47). Stent occlusion was observed in 4 patients. In three cases, it was due to the tumor; an uncovered stent was placed again in these cases. Food-related occlusion developed in one patient. There was no statistical difference in terms of overall adverse event rate when comparing fully covered stents to uncovered stents (*p* = 0.68).

**Conclusion:**

Endoscopic stenting is a viable palliative method with low morbidity and mortality in experienced centers. Though there are relative advantages with covered versus uncovered stents in individual cases, the overall adverse event rate is low and relatively similar.

## 1. Introduction

The number and breadth of endoscopic procedures performed continues to increase. Endoscopy is used universally in the diagnosis and treatment of many diseases. Endoscopic stenting has been increasingly used in the palliation of gastrointestinal malignancies [1]. Stenting provides a relatively easy and effective palliative treatment in patients with metastatic or advanced esophageal cancer.

Endoscopic stenting has been increasingly used in the palliation of gastrointestinal malignancies [1]. Stent insertion provides an easy and effective treatment exclusively in patients with metastatic or advanced esophageal cancer. Endoscopic stenting is a different method for the treatment of anastomosis leakage and esophageal fistula. Stent procedure in distal esophageal malignant stenosis is a simple and uncomplicated treatment method for the patient to relieve correct oral intake and dysphagia [2]. A similar accomplishment is partly achieved in proximal esophageal strictures [3]. Esophageal stent practiced in malignant stenosis can still be successfully practiced in benign stenosis [4]. There are numerous types of self-expandable stents (such as self-expandable biodegradable stents and self-expandable plastic stents). The use of SEMS has been on the increase. Uncovered (UC), semicovered, and fully covered (FC) stents are produced for use in different indications [5]. FC stents are used for anastomotic leakage and fistula. FC stents used for benign diseases can be removed if desired. UC stents are mostly preferred in malignant stenosis. Various complications related to the procedure concur with the use of endoscopic stents. Migration, fistula formation, bleeding, and occlusion are among the most common ones [4].

This study is aimed at discussing the results of self-expandable metal stent (SEMS) applications that we use for palliative treatment in patients with advanced esophageal cancer, in the light of the literature.

## 2. Methods

Study was made in the 1400-bed Necmettin Erbakan University Meram Medical Faculty Hospital in the Central Anatolian region of Turkey. Patients who underwent stenting for palliative treatment in our center due to advanced stage esophageal cancer between January 2014 and June 2019 were evaluated with case series analysis. The research was conducted according to the WMA Declaration of Helsinki-Ethical Principles for Medical Research Involving Human Subjects. The study was approved by the local ethics committee. 60 patients were included in our study. Patients with stent implantation due to benign esophageal stricture and postoperative leakage were excluded from the study. The type of stent was determined according to the indication and localization and size of the lesion. The stent length was determined upon endoscopy. The stent was used in stenoses that did not allow the passage of the scope. In occlusive lesions, the length of the stent was determined by imaging methods adjusting the length of the stent accordingly. We preferred uncovered (UC) stents for tumoral occlusion. Fully covered (FC) stents were preferred for the cases of fistula formation. In our clinic, stents with a length of 10-12 cm and a width of 20 french are used.

All endoscopic procedures were performed by 3 general surgeons in the general surgery clinic. All procedures were performed under anesthesia. The stents were inserted with guidewire under endoscopic control (Figure 1). In cases with in occlusive lesions where the endoscope was inapplicable, dilatation was performed first. 24 hours after the procedure, control radiographs were taken using X-ray. Oral intake was initiated following the X-ray control. Age, gender, location of mass, complications, survival time, and stent type of the patients were evaluated. Both stents (FC and UC) were compared for overall complication, occlusion, and migration development.

### 2.1. Statistical Analysis

The computer software used for biostatistical analysis was Statistical Package for the Social Sciences (SPSS 21 Inc., Chicago, IL, USA). Categorical variables were presented as frequency (percentage), and continuous variables were reported as mean ± standard deviation. Differences in patients' characteristics between FC and UC stents were examined by Pearson's chi-square test for categorical variables.

## 3. Results

Demographic data are given in Table 1. Sixty patients underwent stent insertion. The number of stents was 70. The mean age was 66.4 ± 16. Ten (16%) patients underwent multiple endoscopic stent placement. The stent was successfully inserted in all patients (Figure 1). Oral intake improved in all patients (completely in 75% and partly in 25%, respectively). The mean follow-up period was 133 ± 130 days. The mean length of hospital stay was 2.1 days [1–5].

13 patients developed complications. Migration was the most common complication after stenting. It occurred in 8 (13%) patients who underwent stent placement. In 3 (5%) of these patients, the stent was placed back to its previous position. It was applied especially in patients with migration occurring within a few days. In four (6%) patients, the stents were removed and changed with new ones. Only 1 patient developed a fatal complication. The patient died in the second postoperative month due to mediastinitis due to perforation. Stent migration occurred in 2 patients after chemotherapy (Figure 2). These patients were those who underwent FC stenting due to tracheoesophageal fistula. The old stent was removed, and a new one was placed.

Three patients (5%) developed hypotension during the procedure, and the procedure had to be interrupted. These patients had poor general status and apparent malnutrition. The procedure was successfully performed the next day.

One of the complications related to the stent is occlusion. It was seen in 4 patients. In three cases, occlusion due to a tumor was seen after 3 months. UC stent was placed again in these cases due to tumor growth. Food-related occlusion was observed in one patient and was removed endoscopically. Although the migration rate of FC stents was higher than UC stents, there was no statistically significant difference (*p* = 0.47). There was no statistical difference in terms of complications when FC stents and UC stents were compared (*p* = 0.68) (Table 2).

## 4. Discussion

In both malignant and benign UGI (upper gastrointestinal) tract occlusion, treatment with SEMS is considered to be a safer, less invasive, and effective method than oncological treatments and surgical. SEMS also reduces the rate of complications and length of hospital stay. In recent years, its use has increased as SEMS has a lower morbidity and mortality rate compared to conventional methods [5]. In this study, we shared our SEMS experiences in single center esophageal malignant occlusions. 30% of the cases were located in the proximal esophagus and 70% in the cardioesophageal junction.

While FC SEMS sees more migration, tumor growth is more common in cases with UC stent [6, 7]. We prefer FC stents more frequently due to their complete isolation, particularly in the fistulae, and easy removal. Migration occurred in 4 of 10 cases in which we applied a FC stent. The stents were placed back to their previous position. Stents that fell into the gastric cavity were removed and replaced with new ones. Rarely, stents were fixed with a hemostatic clip.

Most tracheoesophageal fistulas arise from locally advanced malignancy. In such cases, a covered metallic stent is applied for palliative treatment [8, 9]. Fully covered SEMS placement during the early term and minimally invasive drainage is an effective and safe treatment option [10]. In our series, Only 1 patient presented with fatal complications. In the second postoperative month, the patient died because of mediastinitis due to perforation. The occlusion was observed in 4 (6%) cases. They are advantageous as it is easier to remove them once the disease is treated. We mostly preferred FC stents in our cases with fistula formation. The handicap of using this type was a higher rate of migration. Although the migration rate of FC stents was higher than UC stents, there was no statistically significant difference (*p* = 0.47). Consequently, it resulted in a higher number of endoscopic interventions.

Oral intake is corrected in more than 95% of patients undergoing stent insertion due to occlusion [11, 12]. The accomplishment rate in fistula cases changes between 70% and 100% [13]. Stent migration, overgrowth, or ingrowth should be considered in patients presenting with dysphagia after oral intake was previously corrected. Dysphagia was corrected in all of our cases. Occlusion was observed due to tumor ingrowth in three patients. A second stent was inserted to solve these problems. One patient had a food-related occlusion, which was corrected by the endoscopic intervention. Other studies have demonstrated technical success rates (defined as successful insertion and adequate placement of the stent) of 83 to 100% and clinical success rates (defined as palliation of dysphagia) of 80 to 95% ^14.^ In our series, technical success was achieved in SEMS procedures (100%). Dysphagia improved in all our patients. However, 25% of the cases could not tolerate solid food and only tolerated liquid food. Before the stent was placed, all patients had liquid or solid food intolerance. Oral intake was provided after stent placement in all patients.

Although tumor internal growth rates of FC stents are reported to be lower than those of UC stents, migration rates are higher, particularly in the gastroesophageal junction, due to their limited adhesion ability. However, it is reported that short and thinner caliber stents can migrate more. In our series, the stent calibers were the same (20 mm). Stent migration is reported to occur in 10 to 25% of the coated stents and 2 to 5% of the UC stents [14]. The migration rate in our study was 30% in FC stents and 10% in UC stents, and our migration rate was 13% in all cases. Migration rate was higher compared to the literatüre. We think that this situation is caused by the termination of the procedure without waiting for the full opening of the stent during the procedure or the wrong stent selection. Neoadjuvant or palliative chemoradiotherapy is thought to increase the rate of stent migration [15]. Two of our patients had migration after chemoradiotherapy. When FC stents and UC stents were compared, there was no statistically significant difference in terms of complications (*p* = 0.49).

Reocclusion usually occurs as a result of tumor overgrowth or food impaction, and its incidence is reported to be between 3 and 15% for covered and 10 and 42% for uncovered stents [16]. Stents covered with 5-fluorouracil or paclitaxel (drug-eluting stents) have been introduced to prevent tumor ingrowth in recent studies [17]. In this study, food-related occlusion was observed in 1 case and tumor ingrowth occlusion in 3 cases (6%).

Migration, occlusion, perforation, hemorrhage, and ulceration are the most widespread complications related to stents. Mortality rate stent application varies between 0.5% and 2% [ 18, 19]. Complications can be categorized under intraoperative or postoperative complications in the early and late periods. Timing of chemotherapy, stent length, and tumor stage is important parameters in the development of complications [20, 21]. Thirteen of our cases developed complications. Most of them were corrected with small interventions. Mortality was determined as 1%. However, our complication rate is higher compared to the literature. We attributed this situation to the long and strict follow-up period.

## 5. Conclusions

We found that there was no difference between stent types in terms of complication development among patients undergoing palliative endoscopic stenting of advanced esophageal cancers. Endoscopic stenting in this setting has low mortality and morbidity and is effectively in reducing dysphagia. The endoscopist must be experienced and prepared to address complications should they arise.

## Figures and Tables

**Figure 1:** Stent placed in the esophagus.

**Figure 2:** Covered stent migration.

**Table 1:** Demographic characteristics of patients (*n* = 60).

	*n* (patient)	%	Mean ± SD
Sex			
Male	52	86	
Female	8	14	
Age (year)			66.4 ± 16
Survival (month)			4.4 ± 4.3
Stent			
Fully covered	10	16.7	
Uncovered	50	83.3	
Location of mass			
Proximal esophageal ca	18	30	
Cardioesophageal junction tumor	42	70	
Complication			
Migration	8	13	
Occlusion	4	6	
Perforation	1	2	

**Table 2:** Compare of stent types.

	Fully covered stent (*n* = 10)	Uncovered stent (*n* = 50)	*p* value
Complication	4	9	0.68
Migration	3	5	0.47
Occlusion	1	3	0.52

## Data Availability

The data used to support the findings of this study are available from the corresponding author upon request.
